This article has been retracted.

# Real-Time Image Defect Detection System of Cloth Digital Printing Machine

**DOI:** 10.1155/2022/5625945

**Published:** 2022-07-19

**Authors:** Ning Sun, Botao Cao

**Affiliations:** ^1^College of Art and Design, Shaanxi University of Science and Technology, Xi'an, China; ^2^College of Mechanical & Electrical Engineering, Shaanxi University of Science and Technology, Xi'an, China

## Abstract

In order to solve the surface defects such as white silk, spots, and wrinkles on the fabrics in the process of digital printing production, a surface defect detection system for printed fabrics based on the accelerated robust feature algorithm is proposed. The image registration is mainly carried out by the speeded up robust features (SURF) algorithm; the bidirectional unique matching method is used to reduce the mismatch points, realize the accurate registration of the image, and extract the defect information through the difference algorithm. The experiment uses multiple images to verify the performance of the improved SURF algorithm. The experimental results show that the detection accuracy of the new system for surface defects of printed fabrics reaches 98%. The algorithm has higher detection rate and faster detection speed, which can meet the needs of practical industrial applications.

## 1. Introduction

Digital ink-jet printing of fabrics began in the 1990s. It is a high-tech product of the textile industry integrating ink-jet printing technology, computer data processing, and precision instruments [1, 2]. In recent years, with the comprehensive transformation and upgrading of industry, domestic enterprises began to vigorously develop this technology, which played an excellent role in the domestic and foreign markets and made remarkable achievements. However, digital printing technology also has some disadvantages. In the production process, there will be various types of defects in the printing pattern due to nozzle blockage, nozzle ink leakage, cloth wrinkles, motor step deviation, and other faults. In the process of batch printing, if the faults are not found and eliminated in time, a large number of defective products will be produced, resulting in unnecessary waste of resources [3]. At present, although each machine is assigned with corresponding testing personnel, the labor cost is high, the testing standards are not unified, and the human eyes will be tired due to long-time work, so the actual testing effect is not good. Therefore, it is very necessary to develop fast, accurate, and modern industrial testing technology. Image morphological processing is to measure and extract the corresponding shape in the image with certain morphological structural elements, so as to achieve the purpose of analysis and recognition.

In recent years, many scholars have proposed using image processing technology to detect printing defects. Min and Kim proposed a fabric defect detection method based on the Improved Gaussian mixture model, which has a high detection accuracy but does not classify the defect results [4]; Silva et al. proposed a fabric surface defect classification method based on convolutional neural network. This method can classify fabric defects, but its application is limited by application conditions [5]; TZ et al. combined Fourier analysis and wavelet shrinkage and proposed an unsupervised method for detecting fabric defects with periodic patterns. This method simplifies the detection process of periodic fabric defects, but the detection performance is poor [6]; Sachan et al. proposed a detection method to extract the features of the original local binary pattern (LBP) with different resolutions by constructing the Gaussian pyramid model of the printing image. For patterns with complex background textures, this method failed to effectively extract printing defects [7]. Liu et al. proposed a motion texture detection algorithm for Inkjet printing based on a mixed Markov random field model. The algorithm extracts the motion texture features of the image, introduces the mixed Markov model, and constructs a motion texture feature map containing both background state and motion state. After the model is established, the moving texture detection process is transformed into the minimization of feature energy, so as to effectively improve the representation ability of the model for complex textures and improve the accuracy of texture detection [8]. Pennec et al. introduced a textile printing accuracy detection method based on machine vision. Based on the model of a circular screen printing machine, the JSEG algorithm is used to segment the image, find out the edge of the image, match the segmented edge information, and get the deviation region of the image. After experiments, the system has a very good detection accuracy [9]. Khan et al. proposed a dynamic updating method of reference image based on image fusion. Through multichannel differential operation on the image, the defect information is extracted. This method can continuously update and correct the reference image with the industrial production process, but this method is greatly affected by light and noise in the defect detection of printed fabric [10]. Steel and Hartinger proposed a fabric printing color displacement detection method based on normalized cross-correlation. This method mainly matches the image to be measured by moving the standard template and analyzes its differences to determine the color displacement, but this method has high requirements for parameters [11]. An image pyramid is a multiscale representation of an image, an effective but conceptually simple structure for interpreting images at multiple resolutions. An image pyramid of an image is a series of image resolutions that are gradually reduced in a pyramid shape (bottom-up) and originate from the same original image. It is obtained by echelon downsampling and does not stop sampling until a certain termination condition is reached. We liken the image layer by layer to a pyramid. The higher the layer, the smaller the image and the lower the resolution.

## 2. Research Methods

### 2.1. Defect Analysis and Hardware Design of Printed Fabric

#### 2.1.1. Common Printing Fabric Defects

In the process of digital printing production, if the jet printing ink is not filtered thoroughly and contains small particles or motor operation deviation, the nozzle will be blocked; due to mechanical failure of sprinkler head, uneven ink leakage and ink output will be caused; due to the uneven cloth pressing by the roller, there are problems such as cloth wrinkles. The above problems can lead to the surface defects of printing products, such as pass channel, uneven ink output, ink leakage of the nozzle, and cloth wrinkles, and affect the value of the final product [12, 13]. Due to the blockage of the nozzle, uneven ink output of the nozzle, and the deviation of the stepping motor, there are defects such as white silk, spots, and folds in the fabric. See Table 1 for common defect types.

#### 2.1.2. System Hardware Design

Among them, the CCD camera adopts the MVGED501C-T color area array camera of a company, the camera resolution is 1 920 dpi × 1 080 dpi, and the pixel size is 3.45 *μ*m × 3.45 *μ*m. The lighting system adopts LED light source; the lens adopts MV-LD-25-5M-K lens [14]. The schematic diagram of visual platform control is shown in Figure 1.

### 2.2. Surface Defect Detection Algorithm of Printed Fabric

The defect detection function is the core function of the system. In order to realize accurate detection, the defect detection algorithm needs to preprocess the image and extract the characteristic parameters and determine the defect by analyzing the characteristic parameters of the trapped image to be tested and the standard contour image [15, 16]. The software algorithm flow of a defect detection system can be divided into five stages. According to the functional requirements, overall architecture, and data flow direction of the defect detection system, each module cooperates to realize the automatic defect detection function of the system [17].

The surface defect detection algorithm flow of the printed fabric is shown in Figure 2. We carried out the same preprocessing operation for the template image and the image to be detected collected by the camera, use the improved SURF algorithm to match the feature points of the preprocessed image, and affine transform to register the image. After registration, the difference information between the two images is obtained through image difference, that is, defect information.

#### 2.2.1. Image Preprocessing

There is a folder in which several images are placed, and now we classify these images according to their brightness into 10 categories (0–9) and automatically move the images to the corresponding category, which involves the following:

1. Read the Y-U-V value of the image, where the *Y* value represents the brightness of the image
2. File read and write operations in python
3. Use shutil to move files; #The code in this part can refer to the movement of files; it can handle other tasks

Because the collected images of printed fabrics are affected by equipment jitter and insufficient lighting in the factory, problems such as low image brightness, noise, and blurred details affect subsequent operations. Therefore, the collected images need to be preprocessed, and the main processing methods are image grayscale, image contrast enhancement, and image sharpening.

Therefore, the collected images need to be preprocessed. Since the color area array camera used cannot directly obtain the gray image and the color image is not suitable for direct and rapid detection, it is necessary to gray the color image. The steps are as follows [18]:

1. Calculate the RGB component of each pixel of the image
2. Calculate weighted gray value 0.3 × *B* +0.59 × *G* +0.11 × *R*
3. Assign the calculated gray value to each corresponding pixel

Because the collected image has the problem of low brightness, it is necessary to adjust the image contrast to enhance the image. Adjusting image contrast belongs to pixel transformation point operation, and the formula is as follows:

(1) $$\begin{array}{c} g\left(i,j\right)=\alpha f\left(i,j\right)+\beta , \end{array}$$

where *g*(*i*, *j*) is the adjusted pixel; *f*(*i*, *j*) is the pixel before the adjustment; *α* is the gain coefficient, *α*＞0; and *β* is the gain variable.

After the image is grayed and the contrast is adjusted, the image has been significantly improved, but there are some problems such as blurred details, so the image sharpening operation is needed. Image sharpening operations include gradient sharpening and Laplace sharpening. The gradient sharpening effect is good, but the noise resistance is poor. The Laplace method has simple calculation and good real-time performance. Therefore, the research group adopts the Laplace operator to realize image sharpening. The main idea of the sharpening operator is to determine the value of the pixels in the image after traversing Laplace 4.

#### 2.2.2. Image Registration

Due to the placement of the camera and the vibration of the printing equipment, the image to be tested needs to be affine transformed to register the template image for the next defect detection operation. The SURF algorithm uses the approximate image of the Hessian matrix to construct the Hessian matrix of each pixel in the image. When the scale is *σ*, the Hessian matrix of the pixel *X*=(*x*, *y*) is as follows:

(2) $$\begin{array}{c} H\left(x,\sigma \right)=\left[\begin{array}{cc} L_{xx}\left(x,\sigma \right) & L_{xy}\left(x,\sigma \right)\\ L_{xy}\left(x,\sigma \right) & L_{yy}\left(x,\sigma \right) \end{array}\right], \end{array}$$

where *L*_*xx*_ is the second derivative of the filtered image *g*(*σ*) in *x* direction; *L*_*xy*_ is the second derivative of the filtered image *g*(*σ*) in *x* and *y* directions; and *L*_*yy*_ is the second derivative of the filtered image *g*(*σ*) in *y* direction.

Compared with the SIFT algorithm, the SURF algorithm introduces the concept of integral image and uses box filtering with changing size to replace the image pyramid [19]. The response image of the Hessian matrix is obtained by using box filtering and an integral image of each size. In order to select the feature points in the image, the original image needs to be transformed, that is, the approximate value of the Hessian matrix of each pixel in the original image is used to form the transformation image. The weight is introduced to reduce the deviation caused by approximation, and the discriminant is as follows:

(3) $$\begin{array}{c} \text{det}\left(H_{\text{approx }}\right)=L_{xx}L_{yy}-{\left(0.9L_{xy}\right)}^{2}. \end{array}$$

We judge whether the point is a point of interest according to the positive and negative results of (3). The size of the point of interest is compared with the 26 points in its three-dimensional field in the neighborhood of different scale spaces. If the point of interest is the point with the largest eigenvalue in the neighborhood, it is recognized as the feature point in the region.

We take the feature point determined in the previous step as the center, select the area with a radius of 6 S (*s* is the scale value of the feature point), count the Haar wavelet responses of all points in the 60° sector in the area, and give weights according to their responses. The direction of the feature point takes the direction of the longest vector in the area. We take the square box of 20*S∗* 20*S* near the feature point. The box direction is the main direction of the feature point. We divide the box into 4*∗*4 subregions. Each subregion counts the Harr wavelet features of 5*∗*5 pixels. In this way, each subregion has a vector with four-dimensional components. The formula is as follows:

(4) $$\begin{array}{c} V=\left(\sum d_{x},\sum d_{y},\sum \left|d_{x}\right|,\sum \left|d_{y}\right|\right), \end{array}$$

where *d*_*x*_, *d*_*y*_, |*d*_*x*_|, and |*d*_*y*_| represent the sum of horizontal direction and vertical direction and the absolute sum of the horizontal direction and vertical direction, respectively.

So far, each feature point has a 16*∗*4 = 64-dimensional description operator. The Euclidean distance between feature points is calculated to judge whether the matching is correct. The smaller the distance, the higher the similarity. When the Euclidean distance is less than the set threshold, it can be determined that the matching is successful [20].

Affine transformation: although the feature points in the template image and defect image are matched, in practice, the two collected images cannot be fully registered. The transformation parameters need to be determined by matching point pairs to obtain two fully registered images. The schematic diagram of affine transformation is shown in Figure 3.

The affine formula is as follows:

(5) $$\begin{array}{c} \left[\begin{array}{c} m^{\prime }\\ n^{\prime }\\ 1 \end{array}\right]=\left[\begin{array}{ccc} a & b & d_{m}\\ c & d & d_{n}\\ 0 & 0 & 1 \end{array}\right];\left[\begin{array}{c} m\\ n\\ 1 \end{array}\right]=\left[\begin{array}{c} am+bn+d_{m}\\ cm+dn+d_{n}\\ 1 \end{array}\right], \end{array}$$

where (*m*, *n*) and (*m*′, *n*′) are the coordinates of pixels before and after image transformation; *d*_*m*_ and *d*_*n*_ are the translation amounts; and *a*, *b*, *c*,  and *d* are the rotation and stretching parameters.

The matched feature point pair is obtained by the SURF algorithm, and the least square method is selected to fit the matching points to obtain the above parameters. After determining the parameters, we transform according to (5) and finally make the size, position, and angle of the template image and defect image completely consistent.

Neighborhood averaging or weighted averaging can smooth the image, which in turn can sharpen the image using the corresponding differential method. The differential operation is to find the rate of change of the signal, which has the effect of strengthening the high-frequency components so that the outline of the image is clear. Since the essence of image blurring is caused by the average or integral operation of the image, in order to make the edges and blurred contours stretched in any direction clear, inverse operations such as differential operations can be performed on the image to make the image clear.

#### 2.2.3. Defect Detection

After two fully registered images are obtained, the image difference method is selected to obtain the defect location. The basic idea is to differentiate the two images, weaken the similar part of the image, and highlight the changing part [21]. The absolute value of the difference between the gray values of pixels in the same coordinate is taken as the new gray value of the difference image. After the differential operation of the image, the gray value of the defect position will be relatively high, so it will appear white. For the defect-free position, because the pixel values of the two images are the same, the gray value is zero and they appear as black. Because the acquired image is often accompanied by noise and affected by affine parameters during image registration, the difference image often has point or linear “false defects.” After obtaining the above differential image with “false defect,” we carry out image binarization operation and morphological processing to eliminate “false defect” and prominent defect. Morphological processing is used to operate the image information that needs to be highlighted or removed in binary images, including corrosion, expansion, open operation, and close operation. Corrosion reduces the image. Closed operation is usually used to supplement the blank points in the image area.

## 3. Result Analysis

We select the printed fabric with ink leakage defect as the display. Due to the influence of the actual shooting environment, the collected defect map cannot be directly differentiated from the template map. The two images need to be registered after preprocessing [22].

After the matched point coordinate information is obtained, the affine transformation parameters can be obtained by the least square method. We carry out differential operations between the registered defect map and the template map. Due to the different gray values of the template image and the defect image at the defect position, there is an obvious high brightness area at the defect position after the difference and the template image cannot completely coincide due to the influence of affine transformation error. Therefore, there is a ghosting pattern in the difference image. The image is binarized and morphologically operated to eliminate the influence of ghosting and highlight the defect location. The threshold for image binarization is 42, and the structure matrix with a unit structure of 6 × 6 is used for open operation processing. The connected region marking algorithm is used to mark the above point defects, and a rectangular frame with a width of 4 pixels is used to select them. In order to further verify the effectiveness of the detection algorithm of the system, 100 groups of different pictures in the above defect picture library are selected as samples. This algorithm is tested with the traditional template matching method, and the detection accuracy and average value are counted. The results are shown in Table 2.

It can be seen from Figures 4 and 5 that compared with the traditional template matching method, the detection accuracy of the system detection algorithm is 12% higher and the average time is 42.81 ms shorter than the traditional template matching method. Experiments show that the improved SURF algorithm has short time and high precision. The system can meet the actual production needs.

## 4. Conclusion

Aiming at the surface defects of fabrics in the process of digital printing production, as well as the problems of poor real-time performance and low detection accuracy of traditional detection methods, the research group designed a printed fabric surface defect detection system based on an improved SURF algorithm. Compared with the traditional detection algorithm, this algorithm has higher detection rate and faster detection speed and can meet the needs of practical industrial applications.

## Figures and Tables

**Figure 1:** Schematic diagram of the vision platform.

**Figure 2:** Flow chart of surface defect detection.

**Figure 3:** Schematic diagram of an affine transformation.

**Figure 4:** Detection accuracy results of different algorithms.

**Figure 5:** Average detection time results of different algorithms.

**Table 1:** Types of common defects.

Defect type	Reason
Strip and linear	The nozzle is blocked and the ink output of the nozzle is uneven
Lump	Stepping motor deviation and uneven cloth pressing
Punctate	Ink leakage of the nozzle

**Table 2:** Image information table.

Sample	Causes of printing defects	Other algorithms	The algorithm in this paper
Fabric B	6.5336	1.0660	0.1311
Fabric C	5.5351	1.0083	0.4026
Average value	6.0343	1.4821	0.2670

## Data Availability

The data used to support the findings of this study are available from the corresponding author upon request.
